# Impact of parathyroidectomy on cardiovascular outcomes and survival in chronic hemodialysis patients with secondary hyperparathyroidism. A retrospective study of 50 cases prior to the calcimimetics era

**DOI:** 10.1186/1471-2482-13-S2-S4

**Published:** 2013-10-08

**Authors:** Giovanni Conzo, Alessandra F Perna, Vincenzo Savica, Antonietta Palazzo, Cristina Della Pietra, Diego Ingrosso, Ersilia Satta, Giovambattista Capasso, Luigi Santini, Giovanni Docimo

**Affiliations:** 1 Department of Anaesthesiologic, Surgical and Emergency Sciences - VII Division of General and Endocrine Surgery-Second University of Naples - Italy; 2 Department of Cardio-thoracic and Respiratory Sciences - First Division of Nephrology - Second University of Naples - Italy; 3 Papardo Hospital - University of Messina-Italy; 4 Department of Biochemistry and Biophysics “F. Cedrangolo” - Second University of Naples - Italy

**Keywords:** Secondary hyperparathyroidism, parathyroidectomy, parathyroid hormone, cardiovascular outcomes

## Abstract

**Background:**

In chronic hemodialysis patients with secondary hyperparathyroidism, pathological modifications of bone and mineral metabolism increase the risk of cardiovascular morbidity and mortality. Parathyroidectomy, reducing the incidence of cardiovascular events, may improve outcomes; however, its effects on long-term survival are still subject of active research.

We compared, in hemodialysis patients, the results of parathyroidectomy, in terms of cardiovascular outcomes and mortality, with those present in patients following medical treatment only, prior to the diffusion of calcimimetics.

**Methods:**

From January 2004 to December 2006, 30 hemodialysis patients, affected by severe and unresponsive secondary hyperparathyroidism, underwent parathyroidectomy - 15 total parathyroidectomy and 15 total parathyroidectomy + subcutaneous autoimplantation. During a 5-year follow-up, patients did not receive a renal transplantation and were evaluated for biochemical modifications and major cardiovascular events - death, cardiovascular accidents, myocardial infarction and peripheral vascular disease. Results were compared with those obtained in a control group of 20 hemodialysis patients, affected by secondary hyperparathyroidism, and refusing surgical treatment, and following medical treatment only.

**Results:**

The groups were comparable in terms of age, gender, dialysis vintage, and comorbidities. Postoperative cardiovascular events were observed in 18/30 - 54% - surgical patients and in 4/20 - 20%- medical patients, with a mortality rate respectively of 23.3% in the surgical group vs. 15% in the control group. Parathyroidectomy was not associated with a reduced risk of cardiovascular morbidity and survival rate was unaffected by surgical treatment.

**Conclusions:**

In secondary hyperparathyroidism hemodialysis patients affected by severe cardiovascular disease, surgery did not modify cardiovascular morbidity and mortality rates. Therefore, in secondary hyperparathyroidism hemodialysis patients, resistant to medical treatment, only an early indication to calcimimetics, or surgery, in the initial stage of chronic kidney disease - mineral bone disorders, may offer a higher long-term survival. Further studies will be useful to clarify the role of secondary hyperparathyroidism in determining unfavorable cardiovascular outcomes and mortality in hemodialysis population.

## Introduction

Incidence of secondary hyperparathyroidism (2HPT) in the setting of chronic kidney disease-mineral bone disorder (CKD-MBD), increases with dialysis vintage, and, prior to the calcimimetic era, parathyroidectomy (PTx) became necessary in 15% of cases after 10 years, which rose to 38% after 20 years [1]. According to PA Decker et al., an intervention was required in 2.5% of dialysis patients a year [2]. From the analysis of medical treatment results, it emerged that only about half of the patients were controlled in terms of serum calcium (Ca), serum phosphate (P), Ca × P product and intact parathyroid hormone (iPTH)[3]. Recently, calcimimetics, well tolerated allosteric modulators of the calcium-sensing receptor, inhibiting glandular hyperplasia and significantly reducing circulating iPTH levels without exacerbating hyperphosphatemia or hypercalcemia, have been shown to exert a major beneficial impact on 2HTP management. They determine a reduction of fractures, hospitalizations and of PTxs in CKD-MBD population [4,5]. However, R Narayan et al. reported that PTx is more cost effective than cinacalcet in the majority of patients, with the exception of those who are either at high mortality risk, or those who would expect to receive a kidney transplantation in the near future [6]. 2HPT has a negative effect on quality of life under many respects, and induces a higher mortality rate, particularly due to the onset of premature cardiovascular complications, which is associated with vascular calcifications and hypertension. In addition, anemia, at times resistant to erythropoiesis-stimulating agents, becomes a risk factor for unfavorable cardiovascular outcomes [7,8]. The risk for cardiovascular events is increased by 10- to 30-fold among HD patients compared with the general population [9]. It has been demonstrated that at PTH levels > 495 pg/ml there is a 25% increased risk of mortality [10], and the response to vitamin D is reduced by 50% at PTH > 750 pg/ml [11]. Therefore, early surgery could offer an improved quality of life and possibly a higher long-term survival rate. KDIGO parameters modified the National Kidney Foundation (NKF) guidelines [12], by referring to local normal laboratory ranges for Ca, phosphorus and PTH levels, which should be between 2 and 9 times the normal range [13]. Successful surgical treatment often results in a dramatic reduction of iPTH levels, relieving the patient from clinical symptoms [14-17], and different papers showed that PTX could also improve mortality and cardiovascular morbidity [18-23].

With the aim to analyze this issue, we tested the impact of surgery on cardiovascular outcomes and survival in 50 2HPT HD patients, after long-term follow-up. Pre and postoperative cardiovascular status and postoperative outcomes were evaluated in 30 patients submitted to PTx and compared to 20 HD patients refusing surgery. In both populations, calcimimetics were not utilized, and indications to surgical procedure were set according to both K/DOQI 2003 guidelines and Y Tominaga et al. [12,17].

## Materials and methods

### Study design

A retrospective cohort study, in a group of 50 HD patients with severe 2 HPT, unresponsive to medical treatment, selected for PTx, and addressed to our Institution from regional HD centers, was performed. Renal transplantation was considered criteria of exclusion. iPTH levels > 53-84,8 pmol/L, serum P level > 2,09 mmol/l, US enlarged parathyroid glands (> 1 cm or >500 mm^3^) and persisting clinical symptoms, six months after medical therapy, were considered the main criteria for PTx. 30 patients accepted to undergo surgical treatment (surgical group) and 20 patients, refusing surgery, were considered as medical control group. 4 parathyroid glands at least were removed in every case eligible for the study. Cardiovascular disease was defined as presence of hypertension, peripheral artery disease, electrocardiogram (ECG) signs of cardiac hypertrophy, ultrasound (US) cardiac valves calcification, ventricular hypertrophy, arrhythmia, and coronary or cerebrovascular disease. According to P Raggi et al. [24], US valvular calcification was considered as the hallmark of arterial wall calcification in identifying patients affected by severe cardiovascular disease, and an unfavorable prognostic factor, linked to a higher mortality risk. Anemia was evaluated according to the Royal College of Physicians (UK) National Clinical Guideline Centre [25]. During 60 months follow-up, cardiovascular outcomes and survival were evaluated. Mortality data were available trough December 2011. Major cardiovascular events - heart failure, myocardial infarction, peripheral vascular disease and stroke - were the primary end-points, while death was the second end-point.

### Surgical group

Data were retrospectively collected from 30 consecutive patients (11♂ and 19 ♀), affected by 2HPT of CKD, on standard three-weekly HD, and submitted to PTx between January 2004 and January 2006. All patients gave informed consent to participate in the study. Preoperative medical treatment consisted in phosphate chelators (Ca carbonate, sevelamer, lanthanum carbonate), dialysis baths with various Ca concentrations, vitamin D and its analogues. Antihypertensive drugs were used in 22/30 patients (73.3%). The erythropoiesis stimulating agents (ESA) treatment regimen consisted in three-weekly recombinant human ESA (alpha-erythropoietin) injections - 5.200 ± 3824.48 IU, in 29/30 patients. 1/30 patients were treated with alpha darbopoetin 30 (30 μg/every 15 days). Ptx was considered successful when postoperative iPTH level was < 26.52 pmol/L. The 1.06-6.89 pmol/L range was taken as reference of normal iPTH level based on which eu- (1.06-6.89), hypo- (< 1.06), aparathyroidism (0) and persistence or relapse (> 6.89) of disease were determined. Hypocalcemia was considered to be present when serum calcium was <1.99 mmol/L (normal value = 2.09-2.54 mmol/L). High-resolution neck ultrasonography, ear, nose and throat (ENT) examination, technetium- 99m-sestamibi scintigraphy of the neck and mediastinum, were the main preoperative diagnostic procedures. 12-lead ECG and epiaortic 2-dimensional and color doppler transthoracic echocardiogram, by experienced in-center cardiologists, and peripheral artery color doppler ultrasonography examination were pre and postoperatively performed. Cardiac valves calcification was evaluated according to Wong [26]. iPTH, Ca, P, alkaline phosphatase (ALP) and FT_3_, FT_4_, TSH, thyroglobulin were measured along with fine needle biopsy of the thyroid nodules; all blood samples were obtained before dialysis. The Liaison^®^NTact^®^PTH Assay (DiaSorin Inc-Stillwater, MN, USA), based on chemiluminescence immunoassay (CLIA), was used for the quantitative determination of iPTH (Coefficient of variation: CV% intra assay 1.7-3.7; CV% inter assay 2.6-5.9; limit of detection 0.07 pmol/L). Indications to surgical procedure were set according to both K/DOQI 2003 guidelines and Y Tominaga et al. [12,17]. Regarding the surgical procedures, 15 patients underwent total parathyroidectomy (TP) and another 15, awaiting renal transplantation, underwent total parathyroidectomy with autotransplantation (TPai) of 9-15 fragments of non-nodular glandular tissue, in 3 subcutaneous pockets of the non-dominant forearm. In 12 out of 30 patients (40%) with thyroid gland disease, 8 total thyroidectomy and 4 hemithyroidectomy procedures were performed. In all cases, 4 at least parathyroid glands were removed (the nature of the tissue was confirmed via intraoperative histological examination). Only in a few cases, a HD treatment was required immediately after surgery, due to an electrolyte imbalance. The majority of patients required intravenous administration of calcium, due to postoperative hypocalcemia. Patients who underwent autoimplantation completed long-term follow-up monitoring of iPTH from the implantation site and from the contralateral arm, in order to evaluate gradients.

### Medical group

During the same years, 20 patients, (8♂ and 12 ♀), evaluated by a similar preoperative work-up, in which comparable laboratory and clinical criteria for PTx were present (aggressive 2HPT unresponsive to medical therapy), refused surgery for various reasons and were conservatively managed. Medical treatment consisted in phosphate chelators with sevelamer hydrochloride 3200-4000 mg ±1000 in 10/20 (50%) of patients, Vitamin D in 10/20, (50%). Aluminum salts were used in 1 patient and finally calcium carbonate was used in 10 patients. Patients were on three-weekly recombinant human ESA (alpha erythropoietin) injection, 6000 UI in 10/20 patients; 5/20 patients were treated with alpha darbopoietin 60 mcg every week, and 5 with darbopoietin 80 mcg every 15 days. Antihypertensives were used in 60% of patients. Every occurrence of a major cardiovascular event and death was evaluated during a 60 months follow-up.

## Statistics

Data were reported as the mean ± standard error of the mean (SEM). A paired t Student test was performed. The log-rank Mantel-Cox test and the Gehan-Breslow-Wilcoxon test were used to calculate survival. All calculations were performed using the software package GraphPad Prism, Version 5.0 for Windows (GraphPad Software, San Diego, CA, USA). Statistical significance is considered at p < 0.05.

## Results

### Surgical group

#### Demographics

Patient mean age was 51.5 ± 10.89 years, and mean dialysis vintage was 12.93 ± 8 years. Mean preoperative iPTH was 142.08 ± 64.01 pmol/l, and mean serum calcium level was 2.50 ± 0.45 mmol/l (Table 1). All patients reported diffuse pruritus, arthromyalgia and mood alterations, while the incidence of baseline cardiovascular pathologies is reported in Table 2. No case of calciphylaxis was reported. Twelve patients (40%) suffered from coexisting thyroid pathology. None of them had iron deficiency or external blood loss and a mild or moderate anemia (Hb level 7 - <12 gr/dl) was observed (Table 1).

**Table 1:** Characteristics of patients

	Surgical group	Medical group	p value
Age* (years)	51.5 ± 10.89	55 ± 11.20	0.75

Female (%)	63.3	60	n.s.

Dialysis vintage* (years)	12.9 ± 8	10 ± 1.96	n.s.

iPTH* (pmol/L)	142.08 ± 64.01	102.94 ± 32.51	0.03

Ca* (mmol/L)	2.5 ± 0.45	2.4 ± 0,65	n.s.

Anemia (%) (Hb7-<12 gr/dl)**	100	100	n.s.

ESA use (%)	100	100	n.s.

*All data were expressed as mean ± standard deviation; p < 0.05 was considered statistically significant.

**Classification according to the Royal College of Physicians (UK) National Clinical Guideline Centre

ESA = Erythropoiesis-stimulating agent

n.s. = non significant

**Table 2:** Incidence of base-line cardiovascular pathologies (%)

	Surgical group	Medical group
Congestive heart failure	3.3	10

Coronary disease	3.3	10

Myocardial infarction	13.3	5

Cardiac arrhythmias	16.6	-

Peripheral vascular disease	36.6	-

Cardiac valve calcification	33.3	15

### Surgical outcomes

TP and TPai were followed by comparable functional outcomes. Surgical treatment produced a benefit in terms of itching, a substantial improvement in clinical osteoarticular symptoms as well as in mood patterns first, and later in sleep disorders [14-16], an increase in muscular strength, which were associated to a statistically significant reduction in PTH levels (Figure 1), ESA need and improvement of Hb levels. With regard to twelve-months Hb levels, 26/30 pts (86.6%) showed a significant increase and 5 (19.2%) of them had an Hb level >12 gr/dl. No significant variations were reported in 4/30 pts (13.3%).

**Figure 1:** **Preoperative, I° p.o., 1 year and 5 years after surgery mean iPTH levels**. [t test= pre vs I°p.o.: p < 0,05; pre vs 1 year: p < 0,05; pre vs 5 years: p < 0,05]

Regarding the postoperative ESA dosage, 27/30 pts (90%) did not need drug treatment, whilst 3/30 pts (10%) needed a lower dosage. No significant peri- or postoperative complications were observed. None of the patients was found to be aparathyroid (Table 3). Eighteen patients (60%) required intravenous postoperative administration of calcium gluconate due to hypocalcemia, which was occasionally severe, with a minimum value of 1.42 mmol/L, but was never associated with hypocalcemic seizures. The definitive histological examination confirmed the hyperplasia of the removed glands; 2 patients (6.6%) had 5 hyperplastic glands; 8 patients (26.6%) had an associated multinodular goiter, 2 (6.6%) an adenomatous goiter and 2 (6.6%) a papillary carcinoma. Table 3 shows immediate (on postoperative day 1) and long term TP-TPai functional results. After one year, Computed Bone Mineralometry and skeletal x-rays showed a clear regression of osteodystrophy in all patients, irrespective of the procedure carried out. No long-term pathological fractures were reported. In 18/30 patients -54%- postoperative cardiovascular events were observed and mortality rate was 23.3% (Table 4). One patient died for abdominal aortic aneurysm rupture, 3 for congestive hearth failure and 3 for myocardial infarction (after a postoperative mean interval time of 27.2 months). One patient also died for a pulmonary cancer.

**Table 3:** Ptx postoperative results(%)

	Eupara	Hypopara	Persistence	Relapse
I° p.o.	67	20	13	-

1 year	63.3	6	13	17.7

5 years (23pts)	60.9	4.4	13	21.68

Ptx = Parathyroidectomy; Eupara = Euparathyroidism;.

Hypopara= Hypoparathyroidism; I° p.o.: 1 day after Ptx

**Table 4:** Incidence of cardiovascular events and mortality rate during 60 month follow-up (%).

	Surgical group	Medical group
Congestive heart failure	23.3	0

Coronary disease	3.3	0

Myocardial infarction	23.3	10

Cerebrovascular accident	3.3	1

Peripheral vascular disease	6.6	0

Mortality rate	23.3	15

### Medical group

#### Demographics

Patient mean age was 55 ± 11.20 years, and mean dialysis vintage was 10 ± 1.96 years. Mean preoperative iPTH was 102.94 ± 32.51 pmol/l, and mean serum calcium level was 2.4 ± 0,65 mmol/l (Table 1). All patients reported similar clinical symptoms with respect to the surgical group, while cardiovascular disease was found in 20%. Incidence of baseline cardiovascular pathology is reported in Table 2. No case of calciphylaxis was reported. No iron deficiency or external blood loss was observed, while and a mild or moderate anemia (Hb level 7 - <12 gr/dl) was present in every case.

### Outcomes

Pathological fractures were not reported. Cardiovascular events are reported in Table 4. Mortality rate was 15%. Two patients died for cardiovascular disease.

## Discussion

In the present series, PTx did not demonstrate a protective effect against major cardiovascular events, with respect to the incidence observed in the medical control group and also the mortality rate, in patients affected by severe preoperative cardiovascular diseases, was unaffected by surgery (Figure 2), probably because surgery was indicated in 2HPT advanced stages. Even if preoperative iPTH serum levels were higher in surgical patients, the compared groups were similar in 2HPT stage, demographics and preoperative clinical data.

**Figure 2:** **PTx effects on overall survival**. The survival curves relative to the medical control group (dotted line) and PTx group (solid line) are depicted. Months elapsed are plotted against percent survival. The log-rank Mantel-Cox test (p value = 0.5559) and Gehan-Breslow-Wilcoxon test (p value = 0.6592) are not significant for a difference between the two curves.

According to the literature, a lower cardiovascular events-risk was expected in patients undergoing surgery. Dramatic reductions in iPTH serum levels, Ca, P, Ca × P, increase in hematocrit and Hb levels and, possibly, a significant decrease of ESA needs, in most surgical patients, could explain PTx beneficial effects in HD population. In 2HPT of CKD-MBD, pathological modifications of mineral metabolism, particularly phosphate (18), worsening atherosclerosis symptoms and favoring arterial stiffness, increase the risk of cardiovascular morbidity and mortality. Liu et al. reported a high prevalence of CKD-MBD in HD patients with coronary arteries disease diagnosed by coronary angiography [27]. Furthermore, uremia is linked to platelet and coagulation dysfunction [28]. Valvular and arterial wall calcifications, depending on common pathogenetic mechanisms [29], left ventricular hypertrophy and hypertension, are the main unfavorable prognostic factors. Regarding the relationship between cardiac valves calcification and mortality rate, US cardiac valves calcifications were present in 5 of the 7 patients who died in our series. Early surgery could offer a remarkable improvement in the quality of life and, possibly, a higher long-term survival rate. Successful surgical treatment often results in a dramatic reduction of iPTH levels, relieving the patient from clinical symptoms, improving nutritional state and immunity, relieving insomnia and improving cognitive function [14,16,30,31]. Moreover, different papers showed that PTX could also improve mortality and cardiovascular morbidity [18-23]. B Dussol et al. [32] reported that PTx is the main cause of postoperative hypoparathyroidism in HD patients, and is associated with a lower mortality risk, suggesting that a more aggressive 2HPT treatment could decrease mortality. Y Tominaga et al. reported, after PTx, an overall 10-year survival rate of 77.6% in 2000 observed patients [22], higher than that observed in our series (5 years survival of 76.7%). According to the present data, PTx did not demonstrate a protective role against cardiovascular events, and did not modify severe effects of unfavorable vascular uremic ossification. Our results were comparable to those finally reported by EVOLVE Trial [9], demonstrating that, similarly to our surgical trial, calcimimetics likewise did not significantly reduce the risk of death or major cardiovascular events in HD patients affected by moderate-severe 2HPT. Different experimental and clinical studies tried to explain beneficial effects of PTx on cardiovascular outcomes, but they remain unclear [19]. Reductions of iPTH, Ca, P, and increase in serum albumin, hematocrit are the main investigated factors. According to AJ Bleyer et al. [33], PTx may also induce vascular remodeling, but in our series no postoperative regression of cardiovascular calcification was observed. KR Neves et al. [34] suggested that P stimulates the transformation of vascular smooth muscle cells into osteoblast-like cells, creating a promineralization environment. Uremia is associated with a loss of inhibitors of calcification [35] and in addition, parathyroid hormone, acting on vascular system via PTH2 receptors [36,37], may increase atherosclerosis by stimulating vascular smooth muscle cells collagen production [33], or by increasing receptor of advanced glycation end products (RAGE), monocyte-macrophages cytokines and IL-6 expressions [38]. Thus, PTx, with a low morbidity rate similar to that reported in thyroid surgery [39-47], reducing iPTH levels [30], may determine a lower cardiovascular complications rate.

The compared groups were similar in 2HPT stage, demographics and preoperative clinical data, but the relatively small number of examined subjects was the main limitation of this retrospective analysis. Moreover, it must be considered that calcimimetics were not administered; therefore, the impact of novel therapies is not known.

## Conclusions

Our study supports the following: PTx determined a remarkable improvement of quality of life in all cases. However, the lower expected cardiovascular events rate following PTx, compared to that observed in non-surgical patients, was not confirmed. Moreover, mortality was unaffected by surgery, with a 5 years survival of 76.7%. Therefore, a more aggressive multimodal 2HPT treatment should be suggested. Calcimimetics, as well as early surgery, in unresponsive to medical treatment HD patients, may offer an improved quality of life and possibly a higher long-term survival, only if implemented in 2HPT initial stage. Further studies will be useful to clarify the role of 2HPT in determining unfavorable cardiovascular outcomes and mortality in HD population.

## Abbreviations list

2 HPT: secondary hyperparathyroidism; CKD-MBD: chronic Kidney disease-mineral bone disorders; PTx: parathyroidectomy; Ca: calcium; P: serum phosphate; iPTH: intact parathyroid hormone; ECG: electrocardiogram; US: ultrasound; ESA: Erythropoiesis Stimulating Agents; ENT: Ear, Nose and Throat; ALP: alkaline phosphatase; CLIA: chemiluminescence immunoassay; TPai: parathyroidectomy with autotransplantation; SEM: standard error of the mean.

## Competing interests

The authors declare that they have no competing interests.

## Authors' contributions

**GC**: conception, design, and execution of the study; critical revision; analysis and interpretation of data; drafting and editing of the manuscript; given final approval of the version to be published.

**AFP**: conception, design, and execution of the study; analysis and interpretation of data.

**VS**: conception, design, and execution of the study; analysis and interpretation of data.

**AP**: conception, design, and execution of the study; analysis and interpretation of data.

**CDP**: conception, design, and execution of the study; analysis and interpretation of data.

**DI**: conception, design, and execution of the study; analysis and interpretation of data.

**ES**: conception, design, and execution of the study; analysis and interpretation of data.

**GC**: conception and design, given final approval of the version to be published

**LS**: conception and design, given final approval of the version to be published.

**GD**: conception, design, and execution of the study; analysis and interpretation of data; drafting and editing of the manuscript.

## Authors' information

**GC**: Assistant Professor of Surgery at Second University of Naples

**AFP**: Associate Professor of Nephrology at Second University of Naples

**VS**: Associate Professor of Nephrology at University of Messina

**AP**: Surgical fellow at Second University of Naples

**CDP**: Surgical fellow at Second University of Naples

**DI**: Associate Professor of Biochemistry at Second University of Naples

**ES**: Research Fellow in Nephrology at Second University of Naples

**GC**: Full Professor of Nephrology at Second University of Naples

**LS**: Full Professor of Surgery at Second University of Naples

**GD**: Associate Professor of Surgery at Second University of Naples

## Declaration statement

Publication of this article was funded by personal funds.

This article has been published as part of *BMC Surgery *Volume 13 Supplement 2, 2013: Proceedings from the 26th National Congress of the Italian Society of Geriatric Surgery. The full contents of the supplement are available online at http://www.biomedcentral.com/bmcsurg/supplements/13/S2
